# Exploration and Practice of the Integrated Teaching Method of Mind Mapping in the Standardized Training of New Pharmacists

**DOI:** 10.1155/2022/7985027

**Published:** 2022-07-31

**Authors:** Li Yuan, Bei Chen, Zhaojun Wu, Gefei He, Juanjuan Huang

**Affiliations:** Department of Pharmacy, The First Hospital of Changsha, Changsha 410005, China

## Abstract

**Objective:**

The objective is to analyze the application effect of mind map in the standardized training of new pharmacists, providing reference information for the standardized training and teaching methods of new pharmacists.

**Methods:**

24 new pharmacists in pharmacy were selected as experimental samples. The mind map integration teaching method was applied in the standardized training, which involved two parts of pharmaceutical professional knowledge theory and practical skills. The relevant theoretical knowledge of the new pharmacists was evaluated by the examination paper. Their clinical practice ability was evaluated by the expert group on-the-spot assessment score, and the final scores were calculated by two parts. Paired *t*-test was used to analyze the training effect of theoretical knowledge and clinical practice ability of participants before and after training.

**Results:**

All pharmacists have passed the examination. The average score of theory test was (85.8 ± 5.2), the average score of skill examination was (83.1 ± 6.0), and the total score was (84.1 ± 5.0). Before and after training, the total scores of 9 core competencies of pharmacists before and after training have significant difference (18.87 ± 4.06 and 21.40 ± 2.68, *P* < 0.01).

**Conclusion:**

The standardized training for new pharmacists through the mind map integration teaching method can effectively improve their core competence and post competence. This training method is worth using for reference and promotion.

## 1. Introduction

The Development Plan of Medicine and Health points out that the number of hospital pharmacists in China should reach 850,000 by 2020. The standardized training of pharmacists should be strengthened, and the on-the-job training system and professional qualification system of pharmacists should be improved. Pharmacists should be equipped with the relevant policies in hospitals and pharmacies [1]. According to the statistics of China Health Statistical Yearbook 2021, 497,000 pharmacists in medical institutions in China have obtained technical titles by the end of 2020, which is still far from the target of 850,000 pharmacists [2]. In the future, there will be a large number of new pharmacists to enter the hospital. New pharmacists in hospitals refer to pharmacists who have recently graduated or who have obtained the qualification of junior pharmacists within two years. Most of them are fresh graduates lacking practical experience in working in hospitals. It is necessary to change the role of students to pharmaceutical professionals and technicians as soon as possible, to meet the requirements of different positions. It is a new problem for hospital and pharmacy department to strengthen the standardized training of new pharmacists to make them competent pharmacists and to ensure the safety of patients' medication. Standardized training of pharmacists is an important link in the growth of pharmaceutical talents in hospitals, but there has been a lack of standardized system and objective standards for the training of newly recruited pharmacists in our country [3]. At present, a set of effective standardized training course system for new pharmacists has not been formed in China. The notice from the Ministry of Health's Department of Science and Education concerns the implementation in 1999 of standardized training for hospital pharmacists, but the outline did not specify the specific model of standardized training of hospital pharmacists in our country [4]. However, the training model, training objectives, training level, and degree of standardization have not yet reached a unified consensus. Mind mapping integrated teaching method is a new training method, which has been popularized and applied in multi-disciplinary and multi-post staff training. Its training effect has been affirmed by many instructors and participants. In this study, our center combines the mind map integrated teaching method with the standardized training of new pharmacists, taking the new pharmacists in the department of pharmacy as the research object to conduct a systematic theoretical and practical training for a period of 6 months. The training effect is evaluated by the way of examination and assessment, and the experiences and lessons are analyzed and summarized. It can be used as a reference for the further development and system improvement of standardized training for new pharmacists in the later stage.

## 2. Methods

### 2.1. Training Object

In this study, 24 new pharmacists from our center were selected as the research object.

#### 2.1.1. Inclusion Criteria

1. Pharmacists who joined the department of pharmacy or obtained the qualified title of junior pharmacist within 2 years before December 2020 were included in the study;
2. New pharmacists volunteered to participate in this study.

#### 2.1.2. Exclusion Criteria

1. Pharmacists who do not want to cooperate in the research process.

There were six men and 18 women, aged from 21 to 30 years, with an average age of (25.08 ± 2.48), seven have bachelor's degrees and 17 have master's degrees.

### 2.2. Training Mode

Based on the demand-oriented training mode of pharmacists for different positions and paying attention to practical operation, the basic process is shown in Figure 1.

#### 2.2.1. Training Demand Survey

The research group consulted the relevant literature, comping a questionnaire and investigating the students' learning needs for pharmacists with different professional titles before training[5–9]. A total of 1152 pharmaceutical professionals from 99 medical institutions or community health service centers in 13 prefecture-level cities and 1 autonomous prefecture in Hunan Province were selected. 1141 valid questionnaires were collected. The survey shows that the training needs of pharmacists in different positions are different. Pharmacists in outpatient and emergency pharmacies have a strong demand for training in prescription review and rational use of antibiotics, which are closely related to their work. Inpatient pharmacies and static dispensing center pharmacists have a strong demand for training in rational use of antibiotics, rational use of auxiliary drugs, and prescription review due to the use of drugs by patients in all clinical departments of the hospital. Clinical pharmacists need to participate in a series of work, such as pharmaceutical rounds, pharmaceutical consultation, and pharmaceutical consultation. In addition to the basic requirements for pharmaceutical professional knowledge, we also pay more attention to clinical medical knowledge, evidence-based medicine, key case analysis, and case discussion. At the same time, we also observe the demand for medicine and pharmaceutical humanities of pharmacists, which may be related to the change of the demand of the patients for pharmacists. Pharmacists reflect the original intention of changing the pharmaceutical care model. The service is “patient-centered,” and the treatment of patients reflects more humanistic care.

#### 2.2.2. Construct the Detailed Rules for Training Implementation

According to the notice of the Department of Science and Education of the Ministry of Health on the implementation of the standardized training syllabus for Hospital Pharmacists and the Annex “standardized training outline for Hospital Pharmacists” (1999), organize experts to formulate the implementation rules for the training of new pharmacists in our hospital (referred to as “training rules”), including training objectives, implementation objects, curriculum outline, training cycle, training teachers, examination methods, examination standards, and other specific implementation measures.

The training content includes two modules: Professional knowledge and professional skills. The professional knowledge part is the theoretical knowledge training, and the professional skills part is the practical exercise. The specific training courses are shown in Table 1. The purpose of the training is to make hospital pharmacists master the basic knowledge, basic theories, and basic skills necessary for hospital pharmacy. The training of hospital pharmacists should be able to skillfully master the basic knowledge of pharmacy, pharmaceutical-related professional knowledge, laws and regulations, and other comprehensive knowledge. Problem-based teaching method (PBL) or case-based teaching method (CBL) can be adopted in teaching methods. Mind map can be integrated into teaching methods to stimulate the initiative and enthusiasm of new pharmacists.

#### 2.2.3. Implement Training

According to the training implementation rules made in the previous period, the teaching teachers were selected and the training was unified. The training is divided into two stages: the first stage carries on the theoretical centralized training in the online and offline integration mode of the first Hospital in Changsha. The second stage is divided into groups and into different positions of the pharmacy department.

#### 2.2.4. Evaluation and Assessment of Training Effect

Before the implementation of the training, the new pharmacists who participated in the training conducted a theoretical examination. At the end of the training course, they will take part in the theoretical knowledge test and professional skill operation examination. The members of the examination group shall be pharmacists with professional titles in pharmacy and more than 5 years working experience in outpatient and emergency department or hospital adjustment. The examination team formulates the theoretical test paper and the examination standard of skill operation.

1. The total score consists of theoretical and skill scores, of which theory accounts for 40% and skills account for 60%. The main contents of the theoretical examination are the syllabus, the teaching contents of the teachers, and the related knowledge issued by the state, with a total score of 100. Skills assessment uses 4 items of on-site prescription/doctor's order review, drug dispensing, medication account, and simulated patient medication consultation to complete the practice assessment. Each item of the score is 25 points, and the total score is 100 points.
2. Two months after the end of the pharmacist core competence evaluation training, referring to the relevant literature, a self-designed evaluation table was used to evaluate the changes of pharmacist core competence before and after training [10–14]. The scale is evaluated from 9 aspects, including emergency treatment, therapeutic drug testing, adverse reaction report, prescription review, drug storage and maintenance, special drug management, medication guidance and consultation, drug dispensing, and competence in prescription. Basically competent and incompetent are scored, and their weights are 4, 3, 2, and 1, respectively, with a total score of 39 points. Calculating each score and total score, the higher the score, the stronger the pharmaceutical care ability. At the same time, the competency rate is counted and the post competency of the students is evaluated. The calculation formula is as follows: competency rate = competent number + basic competent number/total number.

### 2.3. Statistical Methods

Using SPSS23.0 software, *t*-test was conducted for the score of theory examination, skill operation, and core competence of pharmacists before and after training conforming to normal distribution. *P* < 0.05 or *P* < 0.01 was set as a significant difference, and there was statistical significance.

## 3. Results

### 3.1. Exam Results

All pharmacists have passed the examination, with a pass rate of 100%. The average score of theory test was (85.8 ± 5.2), the average score of skill examination was (83.1 ± 6.0), and the total score was (84.1 ± 5.0). It shows that the trained pharmacists have mastered the basic knowledge and skills of pharmaceutical care. Taking the prescription audit and practical training courses in professional skills upgrading training, new pharmacists draw their own mind maps after training to help memorize knowledge points and operation points as shown in Figure 2.

### 3.2. Comparison of Core Competence Scores of Pharmacists before and after Pharmacist Training

Two months after the training, the score of the pharmacist's core competence is shown in Table 2. After training, the scores of pharmacists' core competence were significantly improved. The total scores of 9 pharmacists' core competence before and after training had significant difference before and after the training (18.87 ± 4.06 vs. 21.40 ± 2.68, *P* < 0.01), indicating that the core competence of pharmacists was significantly improved after training.

The change of post competency of new pharmacists before and after training is shown in Figure 3. The post competency rate of pharmacists was significantly improved after training. Among them, the competencies of emergency management, therapeutic drug monitoring, adverse reaction reports, prescription reviews, drug storage and maintenance, special drug management, drug guidance and consultation, and drug dispensing and prescription/order review increased by 20.84%, 25.00%, 29.17%, 33.33%, 25.00%, 20.83%, 33.34%, 25.00%, and 37.50%, respectively. The prescription/doctor's order review, medication guidance, and consultation and prescription review with low competency rate before training are greatly improved, indicating that the training is highly targeted and meets the job needs of pharmacists.

## 4. Discussion

### 4.1. The Training Mode Dominated by Practical Operation Is Beneficial to Improve the Training Effect

Most of the new pharmacists in the hospital are fresh graduates, lack of practical experience, their knowledge is relatively narrow, and their service skills are relatively weak. They need to change their roles from students to pharmaceutical professionals in order to meet the requirements of different positions. In recent years, after active exploration and practice of standardized training model for hospital pharmacists in many regions and hospitals, Beijing area has initially established a standardized training system for hospital pharmacists in Beijing area. Some hospitals in Shaanxi and Henan have also explored the standardized training model for hospital pharmacists [5, 15–18]. Strengthening the standardized training of new pharmacists, especially in terms of practical skills, is not only an effective way to improve their skills but also an important link to ensure patients' drug safety and improve hospital medical quality and safety. The traditional training mode based on medical and pharmaceutical professional knowledge has played an important role in the early continuing education and standardized training system for pharmacists [19–21]. However, with the increasing requirements of pharmaceutical care and the deepening of rational drug use, pharmacists should not only have solid professional knowledge but also have all-round service skills. A systematic training plan formulated in our center can be targeted to improve the abovementioned skills of new pharmacists and set corresponding assessment standards. Through practical operation, pharmacists can understand their job responsibilities, work contents, system, and standard operating procedures from all aspects, which can not only meet the requirements of pharmacist post competence but also improve the comprehensive quality of pharmacists. The results of this study show that all the trainees passed the examination and the passing rate was 100%. The average score of the theory test was (85.8 ± 5.2), the average score of the skill examination was (83.1 ± 6.0), and the total score was (84.1 ± 5.0). The result shows that the new pharmacists have a high enthusiasm to participate in the training, and they have good participation in the training mode dominated by practical operations. Under this training mode, they can fully stimulate their interest in learning and make them better master the basic knowledge and skills of pharmaceutical care.

The implementation of the practice-led training model for new pharmacists is that the pharmacist team of our hospital fully understands the training programs and needs in different positions and professional titles after detailed investigation in the early stage. The pharmacist training system and model with our characteristics is formed through the careful formulation of the teaching syllabus and training courses by pharmaceutical experts. Through the analysis of the research results, a preliminary understanding of the knowledge reserve of new pharmacists combined with the knowledge and skill requirements of various positions of pharmacists in our hospital. The training courses are reconstructed, the course contents and teaching methods are carefully designed, and the training model of centralized theoretical training and grouping skills practice is implemented. This training model takes pharmacists as the center, following the concept of “teaching according to needs” and paying attention to practical training, and can solve the problems of pertinence and effectiveness of training.

### 4.2. Integrate Various Teaching Methods to Improve the Core Competence of Pharmacists

The results of this study show that after 2 months of theoretical training and skill operation practice, the total scores of the 9 core competencies of new pharmacists are (18.87 ± 4.06) and (21.40 ± 2.68). There was significant difference before and after training (*P* < 0.01), and the post competency rate of pharmacists was significantly improved after training. The competency rates of 9 indicators such as prescription review, drug dispensing, medication guidance, and adverse reaction reports were greatly improved, especially the prescription/doctor's order review, medication guidance, consultation, and prescription review with low qualification rate before training, indicating that the training is highly targeted and meets the job needs of pharmacists.

In the past, the training was mainly based on pharmaceutical theoretical knowledge training, but our training outline was implemented in two stages. In the first stage, centralized theoretical training was carried out in the hospital learning platform in online and offline integration mode. In the second stage, groups were divided into different positions in the pharmacy department for practical training. Theory training had 30 class hours and skills practice had 56 class hours. The total score is composed of theory and skills accounting for 40% and 60%, respectively, which is enough to highlight the new training mode of new pharmacists dominated by skill practice. At the same time, we integrate a variety of effective teaching methods, which could help new pharmacists memorize theoretical knowledge, systematically sort out the knowledge system, and achieve integration [22–24]. Encountering new problems in skills practice, stimulating divergent thinking, and combining practice and theory to form a new mind map deepen the understanding and analysis of theoretical knowledge and gradually adapt to the complex and changeable process of dealing with clinical problems.

At present, our research is mainly limited to Hunan Province with a small number of participants. We will expand our research to the whole China in the follow-up study in order to reduce the limitations of the research.

In conclusion, the implementation of the demand-oriented training model for new pharmacists can grasp the weak links of pharmacists' theories and skills for targeted training, which not only strengthens the skills of rational use of drugs but also enables new pharmacists to have a new understanding of the profession of pharmacists. First of all, the research group has an in-depth understanding of the weak links in the theories and skills of new pharmacists and then formulates well-targeted training rules. At the same time, the integration of various teaching methods is used to improve the core competence of pharmacists, which plays a positive role in improving the level of rational drug use and the construction of pharmaceutical talents.

## Figures and Tables

**Figure 1:** An integrated training model based on the needs of different positions of pharmacists and focusing on practical operation.

**Figure 2:** Mind map of prescription review and practical training points.

**Figure 3:** Comparison of post competency rate of new pharmacists before and after training.

**Table 1:** Outline of training courses for new pharmacists.

Module classification	Professional knowledge (required)	Professional skills (required)	Professionalism (elective)
	Basic knowledge of pharmacy	Capacity of drug supply and allocation	Cultural building
	Professional knowledge related to pharmacy	Pharmaceutical care ability	Moral accomplishment
	Laws and regulations, rules and regulations	Drug management ability	Adaptability
	Drug policy	Interpersonal communication skills	
		Scientific research ability	
		Emergency handling capacity	
School hours	30	56	12
Teaching method	Online and offline integration, centralized training	Group practice (outpatient pharmacy, inpatient pharmacy, pharmacy, and clinical pharmacy)	Online and offline integration, centralized training
Teaching team	Pharmaceutical expert, clinical pharmacist	Senior dispensing pharmacist and clinical pharmacist	Director of pharmacy

**Table 2:** Comparison of core competence scores of pharmacists before and after training.

	Prescription/doctor's order review	Drug dispensing	Medication guidance and consultation	Special drug management	Drug storage and maintenance	Prescription review	Adverse reaction report	Therapeutic drug monitoring	Emergency management
Pretraining score	2.46 ± 0.66	2.79 ± 0.59	2.50 ± 0.66	2.92 ± 0.58	2.75 ± 0.53	2.38 ± 0.65	2.54 ± 0.51	2.63 ± 0.58	2.79 ± 0.59
Score after training	3.08 ± 0.50	3.29 ± 0.55	3.17 ± 0.38	3.46 ± 0.51	3.17 ± 0.48	3.13 ± 0.45	3.00 ± 0.59	3.04 ± 0.46	3.28 ± 0.59
T value	3.668	3.037	4.310	3.425	2.878	4.648	2.890	2.713	2.877
*P* value	<0.01	<0.01	<0.01	<0.01	<0.01	<0.01	<0.01	<0.01	<0.01

## Data Availability

The datasets used and analyzed during the current study are available from the corresponding author upon reasonable request.
